# Study on the Mechanism of Action of Different Acupuncture Regimens on Premature Ovarian Failure Model Rats

**DOI:** 10.1155/2022/5254628

**Published:** 2022-07-25

**Authors:** Yonghao Yuan, Qingchang Xia, Wenzhe Cui, Wen Cao, Ziyang Zhou, Jian Peng, Hailiang Huang, Zhifei Song, Shuying Xie, Runjie Geng, Ran Li, Xiaohua Yu, Jing Zhang

**Affiliations:** ^1^School of Acupuncture and Tuina, Shandong University of Traditional Chinese Medicine, Jinan, Shandong 250355, China; ^2^School of Traditional Chinese Medicine, Shandong University of Traditional Chinese Medicine, Jinan, Shandong 250355, China; ^3^School of Pharmacy, Shandong University of Traditional Chinese Medicine, Jinan, Shandong 250355, China

## Abstract

**Objective:**

To study the mechanism of acupuncture on premature ovarian failure (POF) through the apoptosis pathway mediated by Bcl-2/Bax.

**Methods:**

POF rats were successfully obtained by cyclophosphamide. They were divided into five groups. After that, acupuncture was performed. The blank group and model group were not treated. The routine acupuncture group was acupuncture at Guanyuan, Sanyinjiao, Zhongji, and Guilai four points. The Neck-seven-acupuncture group was selected from Fengchi, Fengfu, Tianzhu, and Wangu four acupoints; the three-viscera simultaneous treatment group selected Guanyuan, Shenshu, Sanyinjiao, Taichong, and Baihui five points; and the data mining group selected Guanyuan and Sanyinjiao two points for 14 days of treatment. During the treatment, some rats were shed one after another due to the side effects of bone marrow suppression caused by mold-making. After treatment, serum estradiol (E2), follicle forming hormone (FSH), and luteinizing hormone (LH) were detected by radioimmunoassay, Bcl-2 and Bax proteins were analyzed by Western blot method, and Bcl-2 and Bax RNA were analyzed by PCR method.

**Results:**

Bcl-2 increased and Bax decreased in rats with premature ovarian failure treated with acupuncture. It shows that acupuncture can affect the secretion of ovarian-related hormones and the expression of apoptosis-related proteins, which is more significant in the conventional acupuncture point group.

**Conclusion:**

Acupuncture can inhibit the apoptosis of granulosa cells in ovarian tissue of rats with premature ovarian failure and improve ovarian function. The mechanism of its effect is to promote Bcl-2 gene expression and protein synthesis and inhibit Bax gene expression and protein synthesis. The conventional treatment group works best. This provides an experimental basis for the clinical use of acupuncture to intervene in the treatment of premature ovarian failure.

## 1. Introduction

Premature ovarian failure (POF) is a general term for a series of symptoms such as amenorrhea before the age of 40 in modern medicine [1]. In ancient China, there was no name of “premature ovarian failure.” According to its performance, it can be classified into categories such as “amenorrhea,” “blood depletion,” and “infertility” [2]. It is a common disease in the field of gynecological endocrinology, with an incidence of 1-3.8% at home and 1% abroad [3]. Premature ovarian failure is characterized by primary or secondary amenorrhea, infertility, low menstrual flow, etc., accompanied by changes in some hormone levels, such as increased blood sex-stimulating hormone (FSH) and decreased estrogen level (E2). At the same time, it will be accompanied by different degrees of symptoms, such as hot flashes, sweating, and facial flushing, which seriously damages the fertility of women of childbearing age and is not conducive to coping with the current pattern of population aging. Generally speaking, the average age of normal amenorrhea in women is 50 to 52 years old, and the age of amenorrhea in patients with premature ovarian failure is much earlier. There are many causes of premature ovarian failure, and the modern and diversified lifestyle further complicates its etiology. Among them, improper weight loss, mental stress, and cold and humid environment, the influence of chemotherapy drugs may cause premature ovarian failure. As a result, premature ovarian failure has become the focus and difficulty of reproductive medicine research. Modern medicine has not made a breakthrough in the prevention and treatment of POF. Hormone replacement therapy has poor efficacy and many side effects, so it is not easy to be accepted by patients [4]. Therefore, it is an urgent problem to seek suitable POF control technology. As a nondrug therapy, acupuncture has fewer side effects and a higher safety factor than the use of hormones. And in the long-term clinical practice, the clinical effect of acupuncture on premature ovarian failure has been fully proved, which has been widely concerned by the medical community. Bcl-2/Bax-mediated apoptosis pathway is involved in the progress of POF. Therefore, this experiment started with Bcl-2/Bax, combined with the data indicators related to the hypothalamic-pituitary-gonadal axis function of endocrine hormones, follicle forming hormone (FSH), luteinizing hormone (LH), etc., to study the mechanism of acupuncture intervention on premature ovarian failure, so as to provide traditional acupuncture technology for treatment. Premature ovarian failure provides new ideas and more reasonable and effective acupoint prescriptions for clinical practice.

## 2. Materials and Methods

### 2.1. Materials

#### 2.1.1. Experimental Animal

There were seventy 8-week-old SPF female Wistar rats (provided by Beijing Weitong Lihua Laboratory Animal Technology Co., Ltd., license number SCXK (Beijing) 2016-0011) with a body weight of 200 ± 20 g. The animals were fed adaptively for a week in the SPF observation room of the Animal Experimental Center of Shandong University of Traditional Chinese Medicine. The room temperature is 22-26°C, and the relative humidity is 60%. Maintain indoor ventilation and natural day and night light.

#### 2.1.2. Experimental Materials and Instruments

Experimental materials and instruments are as follows: sterile acupuncture needle (produced by Suzhou Medical Supplies Co., Ltd., 0.3 mm × 15 mm); cyclophosphamide for injection (Jiangsu Shengdi Pharmaceutical Co., Ltd., product batch number is 18060125); hematoxylin staining solution (Nanchang Yulu Experimental Equipment Co., Ltd., product batch number 181001); 0.9% saline (Shandong Qilu Pharmaceutical Company); methanol, acetone, alcohol, SDS (China Solarbio Co., Ltd., analytical purity); ELISA, Western blot, and PCR kits (China Biyantian Company, UK Abcam Company, US Thermo Fisher Company, US BD Company); 1/10,000 electronic balance (Osho Instruments (Changzhou) Co., Ltd.); microscope (ZEISS Co., Ltd.); ultralow temperature refrigerator and medical refrigerator (China Haier Company); manual micropipette (Germany Eppendorf Company); overspeed centrifuge (Thermo Fisher Company, USA); constant temperature metal bath (Shanghai Jingxin Industrial Development Co., Ltd.); TY-8013 Decolorization Shaker (Jiangsu Science and Technology Instrument Co., Ltd.); cryogenic benchtop centrifuge (Thermo Fisher Company of the United States); automatic water purifier (Millipore Company of the United States); Western blotting vertical electrophoresis apparatus (Bio-PAD, USA); Western blotting transfer membrane apparatus (Bio-PAD, USA); desktop calcium flow detection workstation (American Molecular instrument Co., Ltd.); full-wavelength enzyme labeling instrument (American BioTek Company); multicolor fluorescence imaging system (automatic chemiluminescence gel imaging analysis, American GE Company); ultramicro spectrophotometer (American GE Company); and biochemical incubator (Shanghai Longyue Instrument Equipment Co., Ltd.). The above are used in strict accordance with the instructions.

### 2.2. Experimental Method

#### 2.2.1. Animal Modeling Method

The POF model was prepared by continuous intraperitoneal injection of cyclophosphamide in experimental rats [2]. This method of modeling has a high success rate, is simple and reliable, requires no special apparatus, and is easy to operate. The specific scheme is that after 1 week of adaptive feeding, the rats were fixed in 12 h intervals in the morning and evening twice a day to expose their vaginal opening, and their vulva was first cleaned with a cotton swab dipped in distilled water, after which a cotton swab moistened with saline was slowly inserted into the rat's vagina for 0.8-1 cm and gently rotated and removed, and the secretion was evenly applied to the slide, which was allowed to dry naturally and then fixed with 95% alcohol for 1 min and washed away. The next step was hematoxylin staining for 3 min, followed by washing the slide until there was no hematoxylin discoloration, and after drying, the morphology of rat vaginal cells was observed under a microscope to determine the stage of the animal's motility cycle. From which rats with regular cycles (with an estrous cycle of about 4-5 days, predominantly nucleated epithelium in the preestrous phase, predominantly keratinized epithelium in the estrous phase, predominantly leukocytes in the late estrous phase, and uniform distribution of the three cells in the interestrous phase [2], as shown in Figures 1–4), 7 of the 61 animals were selected by random number table method as blank control group and fed routinely. The rest were modeled by intraperitoneal injection of cyclophosphamide at 8 : 00 every morning for 14 days. The injection dose was 50 mg/kg on the first day and 8 mg/kg every day thereafter [2]. 42 rat POF models were successfully established. The successful rats were randomly divided into model group (without treatment), routine acupuncture group, item seven-needle group, three-viscera cotreatment group, and data mining core acupoint group.

#### 2.2.2. Acupuncture Treatment

After successful modeling, the normal group and model group ate and drank normally and grabbed once a day. The rats in the three Zang-organs treatment group, routine acupuncture group, data mining core acupoint group, and item seven acupuncture group were treated with acupuncture once a day, one day off every six days, and continuous treatment for 14 days. Twist (a TCM acupuncture technique) once every five minutes for one minute each time. The needle is left in place for twenty minutes. The acupoints were positioned by referring to the “Experimental Guidance for Experimental Acupuncture and Moxibustion” combined with anatomy and analogous to the method of measuring the bone size of the human body. Guanyuan was selected in the routine acupuncture group (because the navel of the rats was not obvious after weaning, so the navel was taken as the navel from the xiphoid process to the superior edge of the pubic symphysis, and the downward 25 mm was used to determine the acupoints), Sanyinjiao (the upper 10 mm of the medial malleolus of the hind limb), the middle pole (the intersection of the upper 4 × 5 and the lower 1 pm 5 of the above position of the navel and the upper edge of the pubic symphysis), and return (at the middle extreme level, 5 mm was separated on both sides). For routine disinfection, Guanyuan, Zhongji, and Huilai were injected with 5 mm acupuncture points, and the acupoints on both sides were used for Sanyinjiao and Huilai. In the treatment group, Guanyuan, Shenshu (both sides of the second lumbar vertebra), Sanyinjiao, Taichong (the 1st and 2nd intermetatarsal depressions of the hind limbs of rats), and Baihui (the center of parietal bone) were selected. After routine disinfection, they were treated with stainless steel filiform acupuncture of0.30 × 15 mm, Guanyuan needling 5 mm, twirling and tonifying method. Shenshu needling 2 mm, twirling and tonifying method; Sanyinjiao needling 2 mm, tonifying and reducing method; Taichong needling 1 mm, twirling andreducing method; Baihui needling 1 mm, tonifying and reducing method.Each technique is designed to give a tight feeling under the needle. After the prone position of the rats in the item seven acupuncture group was fixed, the bilateral wind cistern (under the occipital bone, the depression between the upper end of the sternocleidomastoid muscle and the upper end of the trapezius muscle) was obliquely punctured into 5 mm. Fengfu (the back depression of the occipital atlantoid joint behind the occipital ridge), bilateral Tianzhu (beside Fengfu, in the depression of the outer edge of the trapezius muscle), and Wanggu (the depression behind the posterior auricular mastoid) were punctured directly into 3 mm, and the acupuncture was performed with the method of tonifying and relieving. The core acupoint group was determined by data mining, and only two acupoints Guanyuan and Sanyinjiao were selected, and the acupuncture method was the same as the abovementioned acupuncture groups.

#### 2.2.3. Material Method

After the treatment, the rats were weighed. The rats were killed at 60 mg/kg injection using pentobarbital sodium (2% diluted in saline). The blood samples were collected by celiac vein puncture, and the blood samples were placed in 3000 r/min centrifugation 15 min. The supernatant, namely, serum, was stored in the refrigerator at -20°C in the Animal Experimental Center of Shandong University of Traditional Chinese Medicine. Then, disinfect the abdominal skin with ethanol and take aseptic samples. The uterus and ovary on the left side of the abdominal cavity were dissected, cleaned with filter paper, and preserved with liquid nitrogen. After the tissue was precisely weighed, it was placed in the homogenate tube, and normal saline was added in proportion at 1 : 9 to homogenate. The homogenate was placed in EP tube, 3500 r/min centrifugal 15 min, and stored in the negative 80-degree refrigerator on the third floor of the Animal Experimental Center of Shandong University of Traditional Chinese Medicine for follow-up index detection. In the right segment of the uterus and ovary, fat was removed, and after weighing, the ovaries and uterus were immersed in a frozen tube filled with 10% paraformaldehyde solution and fixed.

### 2.3. Detection Method

#### 2.3.1. Analysis of E2, FSH, and LH by ELISA Method

Blood samples were collected by celiac vein puncture; blood samples were placed static and centrifuged, and serum was taken. The contents of E2, FSH, and LH were determined by ELISA kit. According to the principle of double antibody sandwich method, the reagents in the kit were prepared and diluted, and then, the purified antibodies were coated with microwell plates, and the solid phase antibodies were prepared and incubated at 37°C. The antibody-antigen-enzyme-labeled antibody complex was formed by combining it with the labeled antibody. After washing for 5 times, add color developing agent, and finally, convert to yellow after blue color. At this time, adding stop solution, you can measure the absorbance according to the curve and calculate the index concentration according to the difference of color depth, and there is a positive correlation between the two. The entire operation needs to be carried out as soon as possible within 5 minutes to avoid inactivation. After using, it should be stored in the -20°C refrigerator in room 314 of the experimental center. Since room temperature needs to be equilibrated before use, repeated freezing and thawing should be avoided in multiple use projects. Avoid cross-contamination and contact with other irrelevant reagents during the whole process.

#### 2.3.2. Analysis of Bcl-2 and Bax by Western Blot

The protein was extracted from the ice-thawed homogenate of ovarian tissue, and the protein concentration was determined by BCA protein quantitative kit. The parameters for the electrophoretic transfer of the membrane were 150mA steady flow for 2 hours. Prepare 5% nonfat milk powder blocking solution and block overnight, incubate with primary antibody (Bcl-21: 5000, Bax1: 1000, *β*-actin1: 3000) at room temperature for 2 hours, add secondary antibody (1: 2000) for 2 hours, and develop with SuperEclPlus ultrasensitive luminescent solution. X-film was exposed and scanned and processed by the Quantity One gel analysis software, the integral absorbance A of each histone band was measured, and the IA ratio of the target band and the *β*-actin band was used as the expression level of Bcl-2 and Bax proteins.

#### 2.3.3. Determination of mRNA of Bcl-2 and Bax by PCR

Total RNA was extracted from rat ovarian tissues. The purity of total RNA was determined on the basis of absorbance A260/A280, between 1.9 and 2.1, with good purity. And calculate the RNA concentration. Take PCR tube, add the amount of RNA template containing 2 *μ*g as template for reverse transcription, reaction conditions 42°C, hold for 60 min, and inactivate reverse transcriptase by holding at 80°C for 5 min after the end. PCR amplification reaction conditions are as follows: predenaturation at 95°C for 10 min, denaturation at 95°C for 15 s, and extension at 60°C for 1 min, total 40 cycles. The results were sorted by the *ΔΔ*Ct method, and GAPDH was used as the internal reference to calculate the relative mRNA expression levels of Bcl-2 and Bax, which were expressed as 2-*ΔΔ*Ct. The primer sequences are as follows: Bcl-2-F (5′-CTTCGCCGAGATGTCCAG-3′), Bcl-2-R (5′-GGCTCAGATAGGCACCCA-3′); Bax-F (5′-CCCACCAGCTCTGAACAGTTC-3′), Bax-R (5′-CCAGCCACAAAGATGGTCAC-3′); and GAPDH-F (5′-GCACCGTCAAGGCTGAGAAC-3′), GAPDH-R (5′-TGGTGAAGACGCCAGTGGA-3′).

#### 2.3.4. Analysis of the Number of Ovarian Follicles and Corpus Luteum by He Staining on Paraffin Sections

The uterus and ovary of rats were removed, fat was removed, and the ovaries and uterus were immersed in 10% paraformaldehyde solution for fixation, routine sampling, dehydration, paraffin embedding, slice preparation, HE staining, sealing, reading under light microscope, and counting the number of follicles and corpus luteum in the ovary.

#### 2.3.5. SPSS 26.0 Statistical Analysis

The data were analyzed and processed by the SPSS 26.0 statistical software, the measurement data were expressed by *X* ± *S*, the analysis of variance was used for comparison among groups, the LSD method was used for variance, and the Dunnett's T3 method was used for variance discrepancy. Paired *t*-test was used for pairwise comparison, and *p* < 0.05 indicated that the difference was statistically significant.

## 3. Result

### 3.1. Ovarian Index

There was no significant relationship between ovarian index and intervention mode (*p* > 0.05), which may be related to the complex factors affecting the size of ovary (organ mass and body weight of rats are shown in Table 1). And the organ index is generally a toxicological index, which has little to do with the treatment and intervention of premature ovarian failure. The relationship of each group was as follows: neck-seven-acupuncture group > three-viscera simultaneous treatment group > normal group > model group > data mining group > routine acupuncture group; the ovarian index of the three-viscera simultaneous treatment group was similar to that of the normal control group.

### 3.2. Hormone Levels

There were significant differences in the regulation of estrogen in the neck-seven-acupuncture group, follicle-stimulating hormone in the same treatment group, and luteinizing hormone in any group (the sex hormone indicators are shown in Table 2). However, the specific mechanism is not clear, and the hypothalamus and pituitary will be further studied in the future. This is in line with the previous literature that the decrease of FSH and the increase of E2 are more closely related to premature ovarian failure, while the fluctuation of LH may not be closely related to the occurrence and intervention process of premature ovarian failure [5–9].

### 3.3. Bcl-2/Bax

There were significant differences among the groups (the Western blot results are shown in Figure 5, and the PCR results are shown in Table 3). The Bcl-2 mRNA level in the model group was lower than that in the normal group, and the Bcl-2 mRNA level in each treatment group was higher than that in the model group, with the highest level in the conventional acupuncture group. The relationship of each group was as follows: routine acupuncture group > data mining group > three-viscera treatment group > normal group > neck-seven-acupuncture group > model group; three-viscera treatment group and neck-seven-acupuncture group were close to the normal group. Bax mRNA in the model group was higher than that in the normal group, and all treatment groups were lower than those in the model group, among which the routine acupuncture group was the lowest. Routine acupuncture group < data mining group < normal group < three-viscera treatment group < neck-seven-acupuncture group < model group, the three-viscera treatment group was close to the normal group. It can be seen that acupuncture can intervene in the treatment of premature ovarian failure by regulating Bcl-2/Bax. The routine acupuncture group has the best effect, followed by the data mining group. Compared with the routine acupuncture group, more acupoints in the lower abdomen and closer to the surface of the ovary were selected, which may indicate that selecting relevant acupoints will obtain better results [10]. However, there is no significant difference about Bax between theneck-seven-acupuncture group and the model group, which may indicate that neck-seven-acupuncture is not effective for reducing Bax.

### 3.4. Paraffin Section

The number of follicles in each group was lower than that in the normal group, and the number in the model group was the most (the pathological section of ovary in each group is shown in Figure 6, and the number of follicles in each group is shown in Table 4). The three groups of routine group, data mining group, and neck-seven-acupuncture group were all 0, which was significantly different from that of the model group, which may mean that the follicles of the model group stopped developing and remained in the initial stage because of premature ovarian failure. In addition to the model group, the medium-term follicles in each group were more than the normal group, the conventional group was the highest, and the model group was not obvious, indicating that acupuncture has a promoting effect on follicular development. There was no significant difference in the number of late follicles in each group [11–14], but less than the normal group. The number of corpus luteum was significantly different between the conventional group and each group and was less than that of the normal group, and all other groups were more than the normal group. Although the pathological section is the gold standard, the estrous cycle is not differentiated among the groups, and the comparison of the number of follicles and corpus luteum at all levels may lack significance.

## 4. The Rationality of Acupuncture Point Selection

In traditional Chinese medicine, it is believed that the kidney is in charge of reproduction, the liver is in charge of dredging and excretion, it is also in charge of storing blood, and the spleen is in charge of controlling blood, which is closely related to female development. The syndromes of premature ovarian failure in traditional Chinese medicine are also based on this, which is roughly divided into liver-kidney yin deficiency type, heart-kidney noncommunication type, spleen-kidney yang deficiency type, kidney deficiency and liver stagnation type, and kidney deficiency and blood stasis type. Therefore, in terms of syndrome differentiation and treatment, traditional Chinese medicine mainly focuses on restoring the sea of blood, invigorating the kidney qi, regulating the functions of the zang-fu organs, and achieving the purpose of improving symptoms [15]. Based on the analysis of the characteristics and rules of the selection of acupoints in the treatment of infertility by acupuncture and moxibustion in ancient literature, the scheme of simultaneous treatment of three Zang organs pays attention to the selection of acupoints of Ren meridian and foot Shaoyin kidney meridian, highlighting the combined use of acupoints and attaching importance to the application of meridian intersection acupoints, Wushu acupoints, and mu acupoints. The method of selecting acupoints based on syndrome differentiation and syndrome differentiation is emphasized [16]. In the textbook *Acupuncture Therapeutics* of the 13th five-year plan of higher education in the national traditional Chinese medicine industry, the main acupoints for the treatment of amenorrhea are Guanyuan, Zhongji, Sanyinjiao, return, and other acupoints. Guanyuan acupoint is located in Renmai, and it is the intersection of foot Sanyin meridian and Renmai. Zhongji acupoint is located in Renmai, which is the intersection of foot Sanyin and Renmai and the mu acupoint of bladder. Sanyinjiao is located in the foot Taiyin spleen meridian, which is the intersection point of the foot Sanyin meridian. The return acupoint is located in the stomach meridian of foot Yangming, and its name is related to the adjustment of the main function under the menstrual zone. The above acupoints can be used to treat diseases of the female reproductive system. The data mining technology was used to screen the effective literature to find the acupoints with the highest frequency in the effective treatment of premature ovarian failure. The results showed that the most frequently selected meridians were Ren meridian, bladder meridian, spleen meridian, stomach meridian, and kidney meridian, and the most frequently used acupoints were Guanyuan acupoint, Sanyinjiao acupoint, Zusanli acupoint, Shenshu acupoint, and uterus acupoint. To some extent, this also reflects the Chinese medicine in the treatment of syndrome differentiation from the overall point of view, advocating congenital, complementary to make the blood sea restore vitality, so as to improve a series of symptoms of premature ovarian failure. The purpose of this experiment is to study the mechanism of acupuncture on premature ovarian failure model rats, taking into account the experimental process; in line with the concept of complexity and simplicity, select the two most critical points obtained from data mining, and set up the conventional acupuncture group. The results of each group show that acupuncture can change the content of related hormones and proteins and improve the ovarian function of model rats to a certain extent. However, this study has shortcomings; this study is from the rat experimental exploration.There is still controversy about the distribution of acupoints in experimental animals, and their generalizability may be poor. Based on this, we will study the positioning of acupoints in experimental animals in our subsequent work, and strive to be able to extend the experimental findings to the extent that they can guide clinical applications.

## 5. Discussion

A large number of experiments have proved that the content of FSH and E2 in the serum of the core standard animal successfully established by the POF model has changed; that is, the content of FSH is significantly increased, and the content of E2 is significantly decreased. Changes in serum sex hormone levels are important indicators for evaluating ovarian function in POF models. Due to the decrease of serum E2 content caused by pathological low ovarian function, when effective treatment is given and ovarian function gradually recovers, it will naturally rise to close to the normal level, which is an ideal detection index for this experiment. Follicle-stimulating hormone (FSH) can promote the proliferation and differentiation of follicular granulosa cells, tend to mature, and then make the ovary grow. When the ovarian function is damaged, the concentration will increase in feedback and can fall back to the normal level with the recovery of ovarian function, which is a commonly used detection index [17–21]. In this experiment, the above three endocrine hormones are used as reference analysis indicators to judge the success of modeling and the degree of onset of the treatment process. Due to unavoidable cross-reaction and other influencing factors or changes in enzyme activity and pH value due to contamination of impurities and poor storage conditions of tissue samples, some experimental data are also unsatisfactory. At the same time, Bcl-2 (apoptosis inhibitory gene) and Bax (apoptosis promoting gene) were selected as the research indexes at the molecular biological level. Overexpression of Bax can antagonize the inhibitory effect of Bcl-2 and make cells tend to die. Premature ovarian failure is the premature aging of the ovary, and the process of aging is the process of apoptosis. Bcl-2 and Bax were selected as the research indexes on the molecular biological level of apoptosis. Bcl-2 has a decisive role in significantly inhibiting apoptosis, and Bax inhibits the protective effect of Bcl-2 by forming heterodimers and promotes apoptosis. Specifically, in the premature ovarian failure rats modeled by the chemotherapeutic drug cyclophosphamide, Bcl-2 can inhibit ovarian cell apoptosis by enhancing the resistance of cells to DNA damage factors. Although apoptosis may be mediated by some specific pathways, it is not sensitive to Bcl-2/Bax. Or because Bax belongs to Bcl-2 family, both homology, molecular weight, and other properties are close, and Bax expression is far more extensive than Bcl-2, resulting in the impact of experimental data; it may also be due to cross-contamination, primer dimerization, and other factors leading to the accuracy of the experimental results. With regard to the solution of this problem, we will continue to carry out more specific index selection and other related research through network pharmacology analysis in the follow-up plan, follow up the mastery of cutting-edge technology, and strive to get more objective and reasonable experimental conclusions.

In recent years, there have been many studies on the treatment of premature ovarian failure by acupuncture. Kong Suping started from the liver and kidney and took Guanyuan, Sanyinjiao, Taixi, Taichong, and other acupoints, and the research confirmed the rationality of the method of tonifying the kidney and soothing the liver. One of the functional axes of ovarian regulation is hypothalamus-pituitary-ovary axis. Therefore, most scholars believe that acupuncture-related acupoints can stimulate hypothalamus to secrete GnRH, then regulate pituitary gonadotropin secretion, and then regulate ovarian function. The mechanism of premature ovarian failure is not clear. Modern medical treatment believes that premature ovarian failure is closely related to the apoptosis of ovarian granulosa cells. Hormone replacement therapy is often used in clinic. Although this treatment is effective quickly, it is not ideal for the complete recovery of ovarian function. Therefore, some researchers are committed to starting from the root, improve ovarian function to make hormones back to normal, and then make the symptoms of premature ovarian failure disappear. In the field of traditional Chinese medicine, the treatment of related prescriptions has also made great progress, but the specific treatment mechanism is still not clear; the effect of drugs is more complex; different drugs may have different mechanisms. For the time and efficiency of treatment, acupuncture treatment of premature ovarian failure is currently one of the more ideal programs. Several studies have shown that acupuncture can reduce the content of Bcl-2 protein and increase the content of Bax protein, thereby inhibiting ovarian cell apoptosis and improving ovarian function. From the aspect of apoptosis inhibitory genes, the mechanism of premature ovarian failure is also studied on the caspase family and the study on Apaf-1. The above genes, including Bcl family, are the determinants of ovarian granulosa cell apoptosis. Previous studies have shown that endoplasmic reticulum stress proteins can downregulate Bcl-2 and promote cell apoptosis and at the same time lead to the activation of a series of genes related to the caspase family, resulting in cell apoptosis. Related studies have shown that estrogen has an inhibitory effect on endoplasmic reticulum stress proteins. Therefore, we can speculate that the mechanism of acupuncture treatment of premature ovarian failure may be through the upregulation of estrogen and then inhibit the endoplasmic reticulum stress response, so as to achieve the purpose of inhibiting ovarian granulosa cell apoptosis. However, whether other hormones are involved in this regulation process needs further study. In this way, increasing the content of related hormones can indeed improve ovarian function; this regulatory axis forms a closed loop, and the improvement of ovarian function can affect the secretion of related hormones. The mechanism of acupuncture must be more than that, and our hypothesis lays a foundation for further experimental research [22, 23].

In this experiment, the data obtained from the experimental study showed that acupuncture can reduce the FSH content and increase the E2 content in POF model rats and improve the ovarian function of POF rats. However, due to lack of experience in this experiment, there were some inevitable small errors in rat modeling and acupoint positioning. The results of Bcl-2/Bax index were not particularly ideal, but to a certain extent, it proved that acupuncture at acupoints could upregulate the expression of Bcl-2 and inhibit the expression of Bax, thereby inhibiting the apoptosis of ovarian granulosa cells [24–26]. Although there are some omissions in the experiment, after analyzing the problem and finding a feasible solution, it still lays the foundation for our future research. In the future, to further improve the experimental design and carry out more in-depth research on the mechanism of acupuncture in the treatment of premature ovarian failure, it is still expected to provide new ideas and methods for the clinical search for appropriate prevention and treatment techniques for premature ovarian failure [27]. As a clinical practical technology that is easy to learn, promote, and master, it is conducive to solving the technical problems of grass roots and community health service institutions and can further reduce medical costs and improve the quality of medical services [28, 29]. However, this study has shortcomings. At present, the effect and mechanism of electroacupuncture on POF have been explored from the rat level. Clinical experiments need to further confirm the mechanism of electroacupuncture in POF. In addition, the treatment of POF by electroacupuncture involves the Bcl-1/Bax-mediated apoptosis pathway. Whether there are other pathways mediated needs to be further explored in the next experiment.

## 6. Conclusions

In this experiment, POF rat model was built; it was found that Bcl-2 increased and Bax decreased in rats with premature ovarian failure treated with acupuncture. It shows that acupuncture can affect the secretion of ovarian-related hormones and the expression of apoptosis-related proteins, which is more significant in the routine acupuncture group. This indicates that acupuncture can inhibit the apoptosis of granulosa cells in ovarian tissue of rats with premature ovarian failure and improve ovarian function. The mechanism of its effect is to promote Bcl-2 gene expression and protein synthesis and inhibit Bax gene expression and protein synthesis. The routine acupuncture group works best. This provides an experimental basis for the clinical use of acupuncture to intervene in the treatment of premature ovarian failure.

## Figures and Tables

**Figure 1:** Preestrus vaginal smear.

**Figure 2:** Vaginal smear during estrus.

**Figure 3:** Postestrus vaginal smear.

**Figure 4:** Interestrus vaginal smear.

**Figure 5:** Expression of Bcl-2, Bax, and *β*-actin in each group. Note: 85 and 86 are normal groups; 87 and 88 are model groups; 89 and 90 are three-viscera treatment groups; 91 and 92 are seven-needle groups; 93 and 94 are data groups; 95 and 96 are routine groups.

**Figure 6:** (a) Paraffin sections of routine group. (b) Model group paraffin sections. (c) Paraffin sections of the three-viscera treated. (d) Paraffin sections of data mining. (e) Paraffin section of the seven-needle. (f) Paraffin sections of normal. (g) Paraffin section of routine. (h) Paraffin sections of model group. (i) Paraffin sections of three-viscera treated group. (j) Paraffin sections of data mining group. (k) Paraffin section of the seven-needle. (l) Paraffin sections of normal group.

**Table 1:** Ovarian mass, body mass, and ovarian index.

Group	Ovarian weight/mg	Body weight/g	Ovarian index
Normal control group	188.242 ± 36.672	258.000 ± 19.698	1.442 ± 0.294
Model group	180.600 ± 29.715	252.444 ± 10.393	1.427 ± 0.210
Item seven stitches group	168.211 ± 21.626	235.111 ± 22.855	1.537 ± 0.324
Three internal organs treatment group	184.750 ± 16.525	265.125 ± 23.613	1.446 ± 0.191
Data mining group	189.438 ± 29.119	253.625 ± 23.415	1.354 ± 0.143
Routine acupuncture group	183.300 ± 12.056	242.125 ± 20.629	1.323 ± 0.1021

**Table 2:** Difference of hormone levels in each group to the average value of the model group.

Group	E2/(pg/mL)	FSH/(mIU/mL)	LH/(mIU/mL)
Normal control group	0.329687	-0.52283	0.277500
Item seven stitches group	3.659333	-0.377583	-0.441083
Three internal organs treatment group	1.387833	-0.826167	0.006917
Data mining group	0.584625	-0.128083	-1.224937
Routine acupuncture group	0.765875	-0.123458	-1.636062

**Table 3:** mRNA of Bcl-2 and Bax.

Group	Bcl-2	Bax
Normal control group	22.3529 + 0.74651	22.1696 ± 0.82631
Model group	20.1352 ± 0.33802	22.9024 ± 0.26619
Item seven-needle group	20.6405 ± 0.64202	22.7505 ± 0.62806
Three internal organs treatment group	20.9581 ± 0.19195	22.2971 ± 0.26982
Data mining group	21.6252 ± 0.64202	21.6376 ± 0.23624
Routine acupuncture group	22.3529 ± 0.74651	21.1390 ± 0.43992

**Table 4:** Number of follicles and corpus luteum at all levels.

Group	Early follicle (*n*)	Metaphase follicle (*n*)	Late follicle (*n*)	Corpus luteum (*n*)
Normal control group	2.25 ± 2.667	2.08 ± 4.010	0.92 ± 1.240	2.50 ± 1.784
Model group	1.87 ± 1.995	1.67 ± 1.291	0.73 ± 0.884	2.80 ± 3.342
Seven-needle group	0 ± 0	3.07 ± 1.438	0.27 ± 0.458	2.87 ± 1.506
Three internal organs treatment group	1.12 ± 1.799	2.53 ± 1.328	0.65 ± 1.115	3.76 ± 1.348
Data mining group	0 ± 0	2.92 ± 3.095	0.31 ± 0.855	2.85 ± 2.267
Conventional acupuncture group	0 ± 0	3.56 ± 2.007	0.33 ± 0.500	0.44 ± 1.014

## Data Availability

No data were used to support this study.
